This article has been retracted.

# Analysis of the Relevant Vital Signs and Infection of Sepsis Patients and to Explore the Influencing Factors of Acute Lung Injury/Acute Respiratory Distress Syndrome

**DOI:** 10.1155/2022/7718248

**Published:** 2022-09-02

**Authors:** Lei Li, Shida Li, Dong Lan

**Affiliations:** ^1^Emergency Department, Beijing First Integrated Hospital of Traditional Chinese and Western Medicine, Beijing 100026, China; ^2^The First People's Hospital of Guannan, Guannan 223500, China; ^3^Emergency Department, General Hospital of the Western Theater of the Chinese People's Liberation Army, Chengdu 610000, China

## Abstract

In order to analyze the relevant vital signs and infection of sepsis patients, the influencing factors of acute lung injury/acute respiratory distress syndrome (ALI/ARDS) are explored. A total of 142 sepsis patients admitted to our hospital from January 2019 to January 2022 are divided into an ALI/ARDS group and a non-ALI/ARDS group according to the incidence of ALI/ARDS. Logistic analysis showed that pulmonary/abdominal infection, fungal origin of infection, *Acinetobacter baumannii*, low oxygenation index, high blood lactic acid value, APACHE II score, SOFA score, and LIPS score are the risk factors for sepsis-induced ALI/ARDS. The results indicate that pulmonary/abdominal infection, fungal origin of infection, *Acinetobacter baumannii*, low oxygenation index, high blood lactic acid, APACHE II score, SOFA score, and LIPS score are the risk factors for sepsis induced ALI/ARDS.

## 1. Introduction

Acute lung injury/acute respiratory distress syndrome (ALI/ARDS) refers to acute progressive respiratory failure caused by various pathogenic factors other than cardiogenic, trauma, infection, and shock [1]. Acute lung injury and acute respiratory distress syndrome are different stages in the process of the same disease. Acute lung injury represents the early stage of the disease and the condition is mild [2]. Severe acute lung injury is an acute respiratory distress syndrome. The main pathological changes of respiratory distress syndrome are extensive congestion, edema, and hyaline membrane formation in the lungs. The pathological process can be divided into three stages: exudation stage, proliferation stage, and fibrosis stage [3, 4]. Acute respiratory distress syndrome is easy to be complicated with secondary lung infection and form small lung abscess.

Sepsis is prone to cause ALI/ARDS and result in organ dysfunction. In addition, lung injury is the most serious and the first organ with failure symptoms, namely, ALI/ARDS [5]. The current research data show that the incidence rate of ALI/ARDS caused by sepsis is about 24%∼45%, and the mortality of ALI/ARDS patients caused by sepsis is approximately 50%∼60% [6, 7]. The early pathological changes of sepsis are not easy to attract attention and gradually develop into ALI/ARDS. Eventually, it leads to multiple organ failure. At present, protective mechanical ventilation has achieved good therapeutic effect on the disease. However, studies have shown that 40% to 50% of septic patients suffer from ARDS [8]. Once diagnosed with ARDS, patients are often in the serious stage of the disease. Since the pathogenesis of ALI/ARDS has not been accurately understood, the reduction of mortality of ALI/ARDS caused by sepsis has not yet achieved the ideal therapeutic effect [9, 10]. Some studies have pointed out that early diagnosis and timely treatment of sepsis are the key means to combat ALI/ARDS. Therefore, early identification of the risk factors of ALI/ARDS caused by sepsis is of great significance for the treatment of the disease.

The rest of the paper is organized as follows.  Section 2 discusses related studies, and Section 3 introduces the proposed method and observation indicators.  Section 4 describes the results and analysis.  Section 5 provides the summary of the research.

## 2. Related Work

Sepsis is a systemic inflammatory syndrome disease, which can be caused by infection in any part of the body. It has high incidence rate and mortality [11]. Patients with severe sepsis can cause ALI/ARDS, leading to dysfunction of body organs. The direct injury to organ function is lung injury [12]. The clinicopathological manifestation of pulmonary infection is alveolar capillary inflammation, and its pathogenesis is alveolar edema and exudation caused by pulmonary infection. It will lead to alveolar capillary inflammation, which in turn leads to systemic inflammatory response syndrome. Further, ALI/ARDS is induced, which eventually leads to lung function injury [13]. Some studies have shown that pulmonary infection is one of the risk factors for sepsis complicated with ALI [14]. With the popularity of pulmonary artery catheters, ARDS has been proved to be a noncardiogenic pulmonary edema. Later studies further showed that the pathological characteristics of ARDS were increased permeability of alveolar capillary membrane, diffusing lung injury and protein pulmonary alveolar edema. Accompanying physiological abnormalities include severe hypoxemia and decreased lung compliance.

Lung infection and abdominal infection is a sepsis-induced ALI/ARDS factor. If bacterial infection also causes damage to capillaries, severe infection will lead to sepsis and stimulate the body to produce protease and other inflammatory factors. Thus, it will cause a systemic inflammatory response syndrome in the body and ultimately lead to multiple organ function damage, manifested as ALI/ARDS in the lungs [15, 16]. Leopold et al. [17] indicate that the level of oxygenation index is highly correlated with the degree of lung function injury. If the symptoms of ALI are mild, the oxygenation index is high. Liang et al. [18] proposed that in the early stage of sepsis, the lac level in the body will have a high index. The lac level is positively correlated with the severity of ALI/ARDS. Higher lac also leads to increased mortality. The results show that the oxygenation index and blood lactic acid were also the influencing factors of ALI/ARDS caused by sepsis. Leitch et al. [19] showed that with the increase of the APACHE II score, the incidence of ALI/ARDS induced by sepsis also increases, and the mortality of ALI/ARDS patients with severe symptoms also increases. Therefore, the APACHE II score can be used to predict and diagnose the severity of sepsis patients. In addition, the SOFA score [20] can objectively score the degree of multiple organ failure caused by sepsis-induced ALI/ARDS patients and the development degree of ALI/ARDS, which plays an important role in the prediction and diagnosis of ALI/ARDS patients. Sauer et al. [21] have found that LIPS has a good predictive value for ARDS with high reliability. In addition, in this study, it is found that sepsis-induced ALI/ARDS had a higher LIPS score, and the higher the LIPS score, the more serious the lung injury degree. Therefore, it can be concluded that LIPS is a risk factor of sepsis-induced ALI/ARDS. In addition, according to single factor analysis, previous medical history is also a factor that cannot be ignored, so more attention should be paid to such patients, and multiple detection should be conducted to detect the disease as soon as possible and treat it in time [22]. Although certain results have been achieved in this study, there are some shortcomings in this study. Although great progress has been made in the diagnosis and treatment of ALI/ARDS, the diagnosis and treatment of ALI/ARDS is still a challenge for all clinicians and scientists in the field of respiratory diseases. Due to its high mortality, the mechanism of acute respiratory failure and multiple organ failure is not completely clear and the treatment strategy still needs to be improved [23]. Relevant research should be conducted to explore the risk factors of ALI/ARDS induced by sepsis.

## 3. Proposed Method and Observation Indicators

### 3.1. General Information

A total of 142 sepsis patients admitted to our hospital from January 2019 to January 2022 are divided into an ALI/ARDS group (*n* = 82) and a non-ALI/ARDS group (*n* = 60) according to the incidence of ALI/ARDS. ALI/ARDS group included 55 males and 27 females, with an average age of (64.12 ± 12.49) years. The average heart rate is (110.3 ± 21.5) beats/min. The average body temperature is (36.4 ± 1.4)°C. The ALI/ARDS group included 41 males and 19 females, with an average age of (62.44 ± 10.29) years. The heart rate is (109.1 ± 22.1) times/min. The body temperature is (36.5 ± 1.1)°C. There is no statistical significance in age, heart rate, body temperature, and other general data between 2 groups (*P* > 0.05). All the enrolled patients signed informed consent, including that the examination method used in this study is clinically safe. In the process of this study, the original data (including the test sheet) belong to the research group, but we will protect your privacy; no matter when, your name will not appear in the public publications, if the relevant departments need, they have the right to use these data. Your participation is entirely voluntary. You have the right to choose not to participate in this study or to withdraw from it at any time. It does not affect the normal treatment of your disease and your illness, but you hope to complete this study without any special reasons.

The inclusion criteria are as follows: (1) patients who can accept the investigation; (2) meet the diagnostic criteria of sepsis; (3) no other chronic diseases; (4) good understanding and communication skills; and (5) more than 24 hours of admission.

The exclusion criteria are as follows: (1) pregnant women; (2) patients with severe respiratory diseases; (3) patients with cardiac dysfunction and arrhythmia; (4) end-stage patients; and (5) give up treatment of patients.

### 3.2. Proposed Method

The clinical data, infection site, infection agent, and past medical history (such as diabetes, hypertension, and coronary heart disease) of patients in both groups are collected through univariate analysis of the related influencing factors of patients. Clinical data included respiration 24 hours after admission, mean arterial pressure (MAP), heart rate, oxygenation index, acute physiology and chronic health status (APACHE) II score, sepsis-related sequential organ failure (SOFA) score, and blood lactic acid value. Infection sites include lung infection (intrapulmonary/extrapulmonary), abdominal infection, skin infection, urinary system infection, etc. Infection agents included fungi, *Klebsiella pneumoniae*, *Staphylococcus aureus*, and other types of infection agents, as well as lung injury prediction score (LIPS) values in both groups.

The risk factors of ALI/ARDS induced by sepsis are analyzed by multivariate Logistic regression, and the variables with *P* < 0.05 in univariate analysis are put into the multivariate regression model.

### 3.3. Observation Indicators

The observation indicators and evaluation criteria are as follows: (1) Clinical data of patients in the two groups are collected, and the sepsis patient information questionnaire made by our hospital is adopted. Cronbach's coefficient of the questionnaire is 0.84. Including infection site, infection agent, past medical history, respiration 24 hours after admission, mean arterial pressure (MAP), heart rate, oxygenation index, blood lactic acid value, and APACHE II score: including three parts (acute physiological score, age score, and chronic health score). SOFA Evaluation; oxygenation index (PaO2/FiO2): 3002–400 (including 300) is 1 point, 200–300 (including 200) is 2 points, 100–200 needed respiratory support is 3 points, less than 100 needed respiratory support is 4 points, and oxygenation index greater than or equal to 1 point is considered as lung injury. (2) Lung injury is compared between the two groups according to the lung injury prediction score (LIPS) value. High score means serious lung injury. (3) Logistic multiple regression equation is used to analyze the risk factors of ALI/ARDS in sepsis patients.

### 3.4. Statistical Processing

SPSS 24.0 software is used for statistical processing. Measurement data are expressed as mean ± standard deviation (*x*‾±*s*), and comparison between groups is performed with two independent samples *t* test [24]. *χ*^*2*^ test is performed on the count data. Multivariate logistic regression equation is used to analyze the risk factors of ALI/ARDS induced by sepsis patients, and *P* < 0.05 is considered as a statistically significant difference.

## 4. Results and Analysis

### 4.1. Comparison of Past Medical History and Respiration

The patient's past medical history (e.g., diabetes, hypertension, and coronary heart disease) and breathing 24 hours after admission will be compared. The comparison of previous medical history and respiration within 24 h after admission showed a statistical significance (*P* < 0.05). The difference in respiration is not statistically significant (*P* > 0.05) as shown in Table 1.

### 4.2. Comparison of Infection Sites

The incidence of lung and abdominal infection in ALI/ARDS group is significantly higher than that in non-ALI/ARDS group (*P* < 0.05) as shown in Table 2.

### 4.3. Comparison of Infectious Agents

The incidence of infection with fungi and *Acinetobacter baumannii* in ALI/ARDS group is significantly higher than that in non-ALI/ARDS group (*P* < 0.05), as shown in Table 3.

### 4.4. Comparison of Mean Arterial Pressure (MAP), Heart Rate, Oxygenation Index, and Blood Lactate Value

The oxygenation index in ALI/ARDS group is lower than that in the experimental group, and the blood lactic acid value is higher than that in the non-ALI/ARDS group (*P* < 0.05). However, there is no significant difference in other indexes (*P* > 0.05) as shown in Table 4 and Figure 1.

### 4.5. Apache II Score and SOFA Score

APACHE II score and SOFA score in ALI/ARDS group are significantly higher than those in the non-ALI/ARDS group (*P* < 0.05) as shown in Table 5 and Figure 2.

### 4.6. Comparison of Lung Injury Prediction Score (LIPS)

The LIPS score in ALI/ARDS group (6.60 ± 1.50) is significantly higher than that in the non-ALI/ARDS group (3.50 ± 1.40) (*t* = 4.001, *P* = 0.031) as shown in Table 6.

### 4.7. Multifactorial Analysis of Risk Factors for ALI/ARDS in Sepsis Patients

The variables with significant difference *P* < 0.05 in single factor are put into the multifactor regression model for calculation. Pulmonary and abdominal infection, fungal origin of infection, *Acinetobacter baumannii*, low oxygenation index, high blood lactic acid value, APACHE II score, SOFA score, and LIPS score are found to be risk factors for ALI/ARDS in sepsis patients as shown in Table 7.

## 5. Conclusions

In this study, the relevant vital signs and infection of sepsis patients are analyzed and the influencing factors of ALI/ARDS are explored. A total of 142 sepsis patients admitted to our hospital from January 2019 to January 2022 are divided into an ALI/ARDS group and a non-ALI/ARDS group according to the incidence of ALI/ARDS. After univariate and multivariate logistic regression analysis of the two groups of patients, it can be observed that pulmonary and abdominal infection, fungal infection, *Acinetobacter baumannii*, low oxygenation index, high blood lactic acid value, APACHE II score, SOFA score, and LIPS score are the risk factors of ALI/ARDS in sepsis patients. It provides a certain clinical reference for early diagnosis and treatment of sepsis.

## Figures and Tables

**Figure 1:** Comparison of MAP, heart rate, oxygenation index, and blood lactate values.

**Figure 2:** Comparison of the APACHE II score and SOFA score.

**Table 1:** Comparison of past medical history and respiration.

Group	Number	Diabetes (%)	High blood pressure (%)	Coronary heart disease (%)	Breathing 24 hours after admission (%)
ALI/ARDS group	82	44(53.66)	53(64.63)	35(42.68)	24.30 ± 7.30
Non-ALI/ARDS group	60	22(26.67)	26(43.33)	15(25.00)	24.20 ± 8.10
*t/χ* ^*2*^		1.377	2.011	1.147	4.124
*P*		0.045	0.012	0.029	0.054

**Table 2:** Comparison of infection sites.

Group	Number	Lung infection(%)	Abdominal infection (%)	Urinary tract infection(%)	Skin infections(%)
ALI/ARDS group	82	68(82.92%)	53(64.43)	8(9.86)	6(7.31)
Non-ALI/ARDS group	60	34(56.67)	29(48.33)	6(0.10)	7(11.77)
*χ* ^*2*^		4.075	4.413	0.122	0.411
*P*		0.001	0.037	0.051	0.812

**Table 3:** Contrast infectious agents.

Group	Number	*Klebsiella pneumoniae* (%)	*Acinetobacter baumannii* (%)	Fungi (%)	*Staphylococcus aureus* (%)	Others (%)
ALI/ARDS group	82	11(13.41)	44(53.66)	30(37.50)	13(15.85)	23(28.04)
Non-ALI/ARDS group	60	4(6.77)	24(40.00)	15(25.00)	8(13.33)	11(18.33)
*χ* ^2^		2.145	5.413	6.122	1.451	3.412
*P*		0.569	0.002	0.021	0.732	0.055

**Table 4:** Comparison of mean arterial pressure (MAP), heart rate, oxygenation index, and blood lactate values.

Group	Number	Mean arterial pressure (mmHg)	Heart rate (times/min)	Oxygenation index	Blood lactate
ALI/ARDS group	82	81.44 ± 16.24	114.30 ± 21.50	150.50 ± 17.20	5.31 ± 1.03
Non-ALI/ARDS group	60	77.59 ± 14.24	110.60 ± 22.10	175.10 ± 12.50	2.62 ± 1.24
*T*		2.145	5.635	6.122	0.311
*P*		0.569	0.051	0.021	0.032

**Table 5:** Comparison of the APACHE II score and SOFA score.

Group	Number	Apache II score	SOFA score
ALI/ARDS group	82	22.21 ± 6.02	9.82 ± 1.81
Non-ALI/ARDS group	60	15.32 ± 5.23	6.15 ± 1.31
*t*		3.145	3.105
*P*		0.003	0.002

**Table 6:** Comparison of LIPS scores.

Group	Number	LIPS score
ALI/ARDS group	82	6.60 ± 1.50
Non-ALI/ARDS group	60	3.50 ± 1.40
*t*		3.145
*P*		0.003

**Table 7:** Multifactorial analysis of risk factors for ALI/ARDS in sepsis patients.

Factors	*β*	Wald	S.E.	*P*	OR
Lung infection	1.044	1.263	0.349	0.006	4.025(1.331∼5.716)
Abdominal infection	1.203	6.563	0.469	0.001	0.182(0.198∼0.340)
Fungi	0.541	5.513	0.745	0.016	2.105(1.237∼3.198)
*Acinetobacter baumannii*	0.382	5.376	1.081	0.017	0.500(0.579∼1.296)
Oxygenation index	1.001	14.876	0.949	0.003	2.944(1.154∼4.548)
Blood lactic acid value	1.521	13.412	0.413	0.016	3.416(1.224∼3.896)
APACHE II score	0.121	6.745	1.536	0.013	0.112(0.426∼1.452)
SOFA score	0.143	7.856	1.236	0.002	1.458(1.441∼3.741)
LIPS score	1.462	11.762	0.469	0.001	1.897(1.446∼3.446)

## Data Availability

The simulation experiment data used to support the findings of this study are available from the corresponding author upon request.

## References

[1] Briel M., Meade M., Mercat A. (2010). Higher vs lower positive end-expiratory pressure in patients with acute lung injury and acute respiratory distress syndrome: systematic review and meta-analysis. *JAMA*.

[2] Zhou Z. Y., Wang L., Zhang H. L., Liu H. F., Cui Y., Nie H. G. (2020). Participation of mesenchymal stem cells in acute lung injury/acute respiratory distress syndrome: paracrine effects and transplantation. *Science of Advanced Materials*.

[3] Xu B., Chen S. S., Liu M. Z., Gan C. X., Li J. Q., Guo G. H. (2020). Stem cell derived exosomes-based therapy for acute lung injury and acute respiratory distress syndrome: a novel therapeutic strategy. *Life Sciences*.

[4] Fan C. Y., Ding X., Song Y. L. (2021). A new prediction model for acute kidney injury in patients with sepsis. *Annals of Palliative Medicine*.

[5] Li S. L., Zhao D. N., Cui J., Wang L. Z., Ma X. H., Li Y. (2020). Prevalence, potential risk factors and mortality rates of acute respiratory distress syndrome in Chinese patients with sepsis. *Journal of International Medical Research*.

[6] Su L. X., Xu Z., Chang F. X. (2021). Early prediction of mortality, severity, study on the intensity of sepsis in patients with intensive care based on machine learning models. *Frontiers of Medicine*.

[7] Tong M. K., Welten I., Endeman H., Hagenaars T., Ramakers C., Gommers D. (2019). Predicting mortality in adult patients with sepsis in the emergency department by using combinations of Clinical significance of biomarkers for scoring scores: a systematic review. *BMC Emergency Medicine*.

[8] Husabø G., Nilsen R., Flaatten H. (1998). Correction: early diagnosis of sepsis in emergency departments, time to treatment, and association with mortality: an Observational study of an Orchard. *Stomp Lett*.

[9] Al Saleh K., Al Qahtani R. M. (2021). Platelet count patterns and patient outcomes in sepsis at a tertiary care center. *Medicine*.

[10] Hird C. (2020). Early diagnosis and effective management of sepsis. *Nursing Standard*.

[11] Patil N. B., Jotkar S. K. (2020). A Comparative study of quick-SOFA score and serum lactate levels with SOFA score for predicting the clinical outcome in patients with sepsis. *Journal of the Association of Physicians of India*.

[12] Huang M., Cai S. L., Su J. Q. (2019). The pathogenesis of sepsis and potential therapeutic targets. *International Journal of Molecular Sciences*.

[13] Chen H., Liu Q., Wang L. (2018). An analysis of the 28-day mortality risk factors in acute respiratory distress syndrome patients and the Research progress in Translational Science and Technology. *Chinese Journal of Translational Research*.

[14] Lin H., Liang Q., Cai Q., Huang M. (2021). Analysis of high-risk factors and clinical characteristics of sepsis-related liver injury. *Zhonghua wei zhong bing ji jiu yi xue*.

[15] Wang H., Zhao Z., Tong Z. H. (1992). Analysis of risk factors for sepsis and indicators of prognosis in patients with sepsis. *A Retrospective Study of all lands*.

[16] Han S. H., Martin G. S., Maloney J. P. (2011). Short women with severe sepsis-related acute lung injury receive lung protective ventilation less frequently: an observational cohort study. *Critical Care*.

[17] Leopold S. J., Ghose A., Plewes K. A. (2018). Point-of-care lung ultrasound for the detection of Pulmonary infection and sepsis: an experimental study. *Journal of experimental research*.

[18] Liang Y. W., Zhu Y. F., Zhang R. (2019). Incidence, prognosis, and risk factors of sepsis-induced cardiomyopathy. *World Journal of Clinical Cases*.

[19] Leitch A., Wareham D., Melzer M. (2020). Sepsis and the treatment of bacterial infection. *Kumar and Clark’s Clinical Medicine*.

[20] Che U. L., You H. J., Lee J. H. (2020). The index of oxygenation to respiratory rate as a prognostic factor for mortality in Sepsis. *American Journal of Emergency Medicine*.

[21] Sauer C. M., Gomez J., Botella M. R. (2021). Understanding critically ill sepsis patients with normal serum lactate levels - results from U.S. And European ICU cohorts. *American Journal of Respiratory and Critical Care Medicine*.

[22] Lin C. C. (2010). Utility of acute Physiology and chronic health evaluation (Apache II) in predicting mortality in patients A retrospective study of the treatment of abscess of pyogenic liver abscess. *Chinese Journal of Clinical Medicine*.

[23] Li Y. L., Yan C. J., Gan Z. Y. (2019). Prognostic values of SOFA score, QSOFA score and LODS score in patients with Sepsis. *Annals of Palliative Medicine*.

[24] Teng A. K., Wilcox A. B. (2020). A review of predictive analytics solutions for sepsis patients. *Applied Clinical Informatics*.

